The article "Magnetic Resonance Cholangiopancreatography to Evaluate Improvement Effect of FXR Regulating Bile Acid on Hepatocellular Carcinoma with Obstructive Jaundice" was published in 2022. Journal: Contrast Media Mol Imaging.

# Magnetic Resonance Cholangiopancreatography to Evaluate Improvement Effect of FXR Regulating Bile Acid on Hepatocellular Carcinoma with Obstructive Jaundice

**DOI:** 10.1155/2022/3544735

**Published:** 2022-06-23

**Authors:** Liu Wang, Shi Liu, Yuanyuan Li

**Affiliations:** Department of General Surgery, The Third Affiliated Hospital of Qiqihar Medical University, Qiqihar 161000, Heilongjiang, China

## Abstract

This research aimed at exploring the improvement effect of Farnesoid X receptor (FXR) regulating bile acid (BA) on hepatocellular carcinoma with obstructive jaundice under magnetic resonance cholangiopancreatography (MRCP). Forty-eight hepatocellular carcinoma patients with obstructive jaundice who were examined in hospital were selected as the study group, and another 10 healthy volunteers who were examined at the same period were selected as the control group. The patients were treated with FXR inhibitor, and the therapeutic effect was observed. The results showed that after treatment, the AST content and TBIL content in serum of the study group were 123.5 ± 4.9 U/L and 1.8 ± 0.3 *μ*mol/L, respectively, which were significantly lower than those before treatment, *P* *<* 0.05; the ALT content and AST content in serum in patients with high obstruction were significantly lower than those before treatment, and the K^+^ content was significantly higher than that before treatment (*P* *<* 0.05). The ALT, AST, and TBIL contents in serum in patients with low obstruction were significantly lower than those before treatment (*P* *<* 0.05). Apparent diffusion coefficient (ADC) was 1.17 ± 0.49 × 10^−3^ mm^2^/s in patients with moderate jaundice and 1.20 ± 0.27 × 10^−3^ mm^2^/s in patients with severe jaundice, compared with that before treatment, and the difference was statistically significant (*P* *<* 0.05). Based on FXR, it can regulate BA synthesis and metabolism, restore BA metabolic homeostasis, effectively play a hepatoprotective role, reduce bilirubin content in the body, and improve jaundice injury, which has application value.

## 1. Introduction

Hepatocellular carcinoma with obstructive jaundice is defined as obstruction of bile excretion and cholestasis due to invasion or compression of the hepatobiliary duct or common bile duct by various direct or indirect causes, which is clinically characterized by hyperbilirubinemia, yellow staining of tissues or body fluids, and bile duct dilatation [1]. Obstructive jaundice can be divided into benign and malignant obstructive jaundice [2]. The hilar bile duct is often used as the demarcation line for the two, and the causes of obstruction can be direct compression of the bile duct by the primary tumor around the liver, gallbladder, bile duct, pancreas, and ampulla, or obstruction caused by tumor metastasis invading the bile duct at other sites [3]. The core problem of jaundice damage to the body is a series of organ dysfunctions with liver damage as the source caused by persistent and progressive obstruction of the biliary tract. Persistent obstruction makes bile unable to enter the intestine normally, and a large amount of bilirubin stasis in the liver, and then a large amount of bilirubin into the blood, forming hyperbilirubinemia, at this time with the impact of malignant tumors, so that the body produces a series of pathophysiological disorders [4]. Relevant studies have shown that degeneration, necrosis, and intrahepatic cholestasis occur in hepatocytes when bile duct obstruction occurs for 3 to 5 days, and with the persistence of bile duct obstruction, bile canalicular proliferation, fibrosis, and even biliary cirrhosis occur [5].

The article "Magnetic Resonance Cholangiopancreatography to Evaluate Improvement Effect of FXR Regulating Bile Acid on Hepatocellular Carcinoma with Obstructive Jaundice" was published in 2022. Journal: Contrast Media Mol Imaging.

Imaging examinations such as ultrasound, CT, MRI, and endoscopic retrograde cholangiopancreatography (ERCP) are used for the diagnosis and differential diagnosis of calculous obstructive jaundice, especially magnetic resonance imaging (MRI) has been widely used for the detection and characterization of liver lesions, and the evaluation of tumor treatment effects [6]. Magnetic resonance cholangiopancreatography (MRCP) can clearly show the location of obstruction and the number of stones, but it can only provide morphological information of the liver and biliary system, but cannot reflect the functional status of the liver. Because liver dysfunction caused by persistent cholestasis is an important manifestation of obstructive jaundice, the evaluation of liver function in clinical practice is mainly through serum biochemical monitoring [7–9]: (1) protein metabolic function monitoring; (2) plasma coagulation factor determination; (3) serum bilirubin determination, which is an important indicator to assess the degree of jaundice; (4) bile acid (BA) metabolism detection, which is synthesized by cholesterol in the liver, and the determination of which can reflect the synthesis, uptake, and secretion function of hepatocytes, and is related to biliary excretion function; (5) liver function test, indocyanine green (ICG) retention test; and (6) detection of serum enzymes and isoenzymes.

BAs are a general term for a large group of cholanic acids found in bile. As the main component of bile, they often exist in the form of sodium or potassium, which is called bile salt [10]. The BAs are to form mixed micelles through the characteristics of their surfactants to promote the dissolution, digestion, and absorption of fat and fat-soluble vitamins; it can also maintain the homeostasis of cholesterol in the body by promoting the absorption of intestinal nutrients and the secretion of cholesterol in bile, thereby protecting the liver and other tissue cells from the toxicity of high cholesterol; it can protect the intestine, remove endotoxin, act as a chemical barrier of the intestinal mucosa, and maintain the stability of the intestinal microbiome under normal physiological conditions, and most BAs have a significant antibacterial effect on *Staphylococcus aureus* and *Escherichia coli* [11]. In recent years, through the study of BA metabolism, it has been found that BA is not only an energy-derived substance in the body, but also an important signaling molecule, which is involved in the regulation of glucose and lipid metabolism, energy metabolism, and inflammation in the enterohepatic circulation system and peripheral organs by activating different signaling pathways [12].

The article "Magnetic Resonance Cholangiopancreatography to Evaluate Improvement Effect of FXR Regulating Bile Acid on Hepatocellular Carcinoma with Obstructive Jaundice" was published in 2022. Journal: Contrast Media Mol Imaging.

With the in-depth study of metabolism, scholars have found that in addition to the general physiological function of BA metabolism, it can also indirectly regulate many biological processes of the body. When the homeostasis of BA metabolism in the brain-enterohepatic axis is destroyed, it can cause a series of diseases, which are closely related to the hepatobiliary system, nervous system, etc. It has become a research hotspot in liver disease, encephalopathy, metabolic diseases, etc. [13]. Nuclear receptor Farnesoid X receptor (FXR) is the most important receptor that controls BA metabolism and is involved in affecting the enterohepatic circulation system. By regulating the expression of related key enzymes and target genes, FXR is involved in the regulation of BA synthesis, efflux, metabolism, intake, and transport, which is of great significance for reducing the toxicity of BAs to the liver, maintaining the homeostasis of BAs, maintaining body homeostasis, and exerting a protective effect on the liver [14]. FXR is widely distributed in various tissues such as liver, intestine, adipose tissue, vascular wall, pancreas, and kidney, especially highly expressed in tissues and organs closely related to BA metabolism such as liver and intestine, which can regulate the absorption, metabolism, and secretion of BAs [15].

Therefore, patients with obstructive jaundice due to liver cancer were selected as the study subjects to regulate BA changes in patients by FXR inhibitor treatment and to observe its therapeutic effect on obstructive jaundice injury with the help of MRI cholangiopancreatography. It provides data and theoretical support for the evaluation of the therapeutic effect of obstructive jaundice injury in liver cancer in the future clinical practice.

The article "Magnetic Resonance Cholangiopancreatography to Evaluate Improvement Effect of FXR Regulating Bile Acid on Hepatocellular Carcinoma with Obstructive Jaundice" was published in 2022. Journal: Contrast Media Mol Imaging.

## 2. Research Methods

### 2.1. Study Subjects

Forty-eight hepatocellular carcinoma patients with obstructive jaundice who were examined in hospital from January 2019 to June 2021 were selected as the study group, including 20 males and 28 females, with an average age of 52.61 ± 9.59 years. All patients were treated with FXR inhibitors and could be classified according to the serum bilirubin content as mild jaundice: 34–170 *μ*mmol/L, moderate jaundice: 170–240 *μ*mmol/L, and severe jaundice: >340 *μ*mmol/L. According to the site of obstruction, it was divided into high obstruction and low obstruction. Another 10 healthy volunteers examined in the Hospital during the same period were selected as the control group, including 5 males and 5 females, with a mean age of 46.74 ± 7.92 years. The families of the patients signed the informed consent form, and the trial process was approved by the ethics committee of hospital.

Inclusion criteria are as follows: (1) biochemical tests suggested elevated serum bilirubin; (2) imaging diagnosis showed benign intrahepatic and/or extrahepatic bile duct stone obstruction; (3) intrahepatic or extrahepatic bile duct stones confirmed by surgery; and (4) liver cancer confirmed by pathological examination. Exclusion criteria are as follows: patients with other chronic liver diseases.

### 2.2. Detection of Total Bile Acid (TBA) Level

Blood samples were collected from veins in the morning (fasting), and serum was separated and placed at 20°C for examination. Basic principle: the level of TBA was determined by the double antibody sandwich method. The extracted TBA was added into the micropores of the coated monoclonal antibody and combined with the HRP-labeled TBA body to form an antibody-antigen-enzyme-labeled antibody complex. After thorough washing, the substrate TMB was added for color development. TMB changed from blue to yellow under the catalysis of HRP and acid, and the color depth was positively correlated with the TBA content in the sample. The OD value was measured at 450 nm by enzyme labeling instrument, and the concentration of TBA in the sample was calculated by the established TBA standard curve [16].

### 2.3. Upper Abdominal MRI and Laboratory Tests for Liver Function

3.0 T magnetic resonance scanner was used. Each patient was fasted for 6–8 hours before the examination, and the patient's breathing was trained before the scan, so that the patient can better cooperate with the breath-holding. Routine MRI scanning was performed in the supine, head-forward position, the upper abdomen was surrounded by an abdominal phase-controlled display coil, and routine T1WI, T2WI, coronal T2, and MRCP scans of the liver were performed. DWI examination was performed with the body coil as the radiofrequency transmit coil and receive coil, using the SE-EPI sequence and prospective acquisition correction (PACE), axial, TR: 5,900 ms, TE: 83 ms, slice thickness: 6.59 mm, interval: 1 mm, field of view: 284 × 376 mm, matrix: 115 × 192, NEX = 1. The *b* value (diffusion-sensitive gradient coefficient) was taken as 50, 400, and 800 s/mm^2^.

The article "Magnetic Resonance Cholangiopancreatography to Evaluate Improvement Effect of FXR Regulating Bile Acid on Hepatocellular Carcinoma with Obstructive Jaundice" was published in 2022. Journal: Contrast Media Mol Imaging.

All MRDWI images automatically generated apparent diffusion coefficient (ADC) maps by magnetic resonance postprocessing workstation, and two experienced MRI diagnostic experts jointly evaluated the image quality and measured the ADC values of the liver in the qualified scanning images. Since the left lobe of the liver was susceptible to cardiac motion, the circular region of interest (ROI) for measuring the ADC value of the liver parenchyma was located at the level near the hilum of the right lobe of the liver, with each circular ROI area of 79 mm^2^ (1 cm in diameter), which contained about 776 voxels, and the visible hepatic vasculature should be avoided as much as possible during measurement.

The laboratory examination of the liver function of all patients was to draw 5 mL blood from elbow vein when fasting and analyze it automatically by the Beckman Coulters automatic biochemical instrument; the time between laboratory examination and MRI examination was less than 48 hours. Laboratory test indicators included alanine aminotransferase (ALT), aspartate aminotransferase (AST), serum total bilirubin (TBIL), and electrolytes (Na^+^, K^+^).

### 2.4. Statistical Methods

SPSS 22.0 statistical software was used for data management and statistical analysis. Measurement data were expressed as mean ± standard deviation, means were compared using the *t*-test, and categorical variables were compared using *x*^2^ test, with *P* *<* 0.05 considered statistically significant.

## 3. Results

### 3.1. General Information

Fifty-eight subjects were included, including 25 males and 33 females. After examination, there were 26 cases of high biliary obstruction and 22 cases of low biliary obstruction; There were 8 cases of mild jaundice, 24 cases of moderate jaundice, and 16 cases of severe jaundice (Table 1 and Figure 1).

### 3.2. Changes in BA Levels

The detection results of serum TBA showed that the content of serum TBA was 13.5 ± 0.4 mmol/L and intrahepatic TBA was 34.6 ± 0.6 mmol/L in the control group. The serum TBA was 11.2 ± 0.6 mmol/L, and intrahepatic TBA was 12.4 ± 1.8 mmol/L in the study group before treatment. Compared with the control group, the content in the study group decreased significantly, and the difference was statistically significant (*P* *<* 0.05). After treatment, the content of serum TBA and intrahepatic TBA in the study group were 12.8 ± 0.5 mmol/L and 28.3 ± 1.2 mmol/L, which increased significantly compared with that before treatment, with a statistically significant difference (*P* *<* 0.05). Although there was a difference compared with the control group, it was not significant, *P* *>* 0.05 (Figures 2 and 3).

The article "Magnetic Resonance Cholangiopancreatography to Evaluate Improvement Effect of FXR Regulating Bile Acid on Hepatocellular Carcinoma with Obstructive Jaundice" was published in 2022. Journal: Contrast Media Mol Imaging.

### 3.3. Laboratory Test Results

The contents of AST, ALT, TBIL, Na^+^, and K^+^ in the serum of the control group were 118.4 ± 6.2 U/L, 55.7 ± 1.2 U/L, 1.9 ± 0.4 *μ*mol/L, 135.74 ± 4.76 mmol/L, and 4.14 ± 0.52 mmol/L, respectively; before treatment, the content of AST in the serum of the study group was 146.3 ± 9.7 U/L, which was significantly higher than that of the control group, and the difference was statistically significant (*P* *<* 0.05). Although other contents increased or decreased in varying degrees, the difference was not statistically significant (*P* *>* 0.05). After treatment, the content of AST in serum was 123.5 ± 4.9 U/L, which was significantly lower than that before treatment, *P* *<* 0.05. The content of TBIL was 1.8 ± 0.3 *μ*mol/L, which was significantly lower than that (2.2 ± 0.5 *μ*mol/L) before treatment, *P* *<* 0.05. There was no significant change in other contents (Figure 4).

### 3.4. Changes of Liver Function at Different Obstruction Sites

The detection results of the changes in liver function in patients with obstruction at different sites showed that after treatment, the serum ALT content of 55.7 ± 31.6 U/L, AST content of 66.4 ± 42.4 U/L, and TBIL content of 215.4 ± 136.32 *μ*mol/L in patients with high obstruction were significantly decreased compared with those before treatment, and the differences had statistical significance (*P* *<* 0.05); the K^+^ content of 4.13 ± 0.4 mmol/L was significantly increased compared with that before treatment, and the difference had statistical significance (*P* *<* 0.05) (Figure 5). The serum ALT content of 47.4 ± 32.8 U/L, AST content of 56.1 ± 25.9 U/L, and TBIL content of 142.5 ± 123.6 *μ*mol/L in patients with low obstruction were significantly decreased compared with those before treatment, and the differences were statistically significant, *P* *<* 0.05 (Figure 6).

### 3.5. MRI Test Results

The results of MRI showed that ADC was 1.34 ± 0.32 × 10^−3^ mm^2^/s in the control group, 1.24 ± 0.44 × 10^−3^ mm^2^/s in patients with mild jaundice before treatment, 1.18 ± 0.67 × 10^−3^ mm^2^/s in patients with moderate jaundice, and 1.02 ± 0.66 × 10^−3^ mm^2^/s in patients with severe jaundice; compared with the control group, the difference was statistically significant (*P* *<* 0.05); ADC was 1.17 ± 0.49 × 10^−3^ mm^2^/s in patients with moderate jaundice and 1.20 ± 0.27 × 10^−3^ mm^2^/s in patients with severe jaundice after treatment; compared with that before treatment, the difference was statistically significant (*P* *<* 0.05). Although ADC values were slightly increased in patients with mild jaundice, compared with those before treatment, the difference was not statistically significant (*P* *>* 0.05) (Figure 7).

The article "Magnetic Resonance Cholangiopancreatography to Evaluate Improvement Effect of FXR Regulating Bile Acid on Hepatocellular Carcinoma with Obstructive Jaundice" was published in 2022. Journal: Contrast Media Mol Imaging.

## 4. Discussion

FXR regulates the synthesis of BAs in a tissue-specific manner. High levels of ligands activate the expression of hepatic FXR. FXR inhibits the synthesis of BAs in the classical pathway by inducing the expression of target gene atypical nuclear receptor small heterodimer partner (SHP) and further inhibiting the expression of rate limiting enzyme CYP7A1. The inhibition of the classical pathway often feeds back the activation of alternative pathway synthase [17]. The results of serum TBA content detection in patients with hepatocellular carcinoma and obstructive jaundice treated with FXR inhibitor showed that the serum TBA content was 13.5 ± 0.4 mmol/L and the intrahepatic TBA content was 34.6 ± 0.6 mmol/L in the control group. The serum TBA content was 11.2 ± 0.6 mmol/L, and the intrahepatic TBA content was 12.4 ± 1.8 mmol/L before treatment in the study group, which was significantly decreased compared with the control group, and the difference had statistical significance (*P* *<* 0.05); the serum TBA content was 12.8 ± 0.5 mmol/L, and the intrahepatic TBA content was 28.3 ± 1.2 mmol/L after treatment in the study group, which was significantly increased compared with that before treatment, and the difference had statistical significance (*P* *<* 0.05). Studies have shown that liver injury causes BA intestinal and hepatic circulation disorders and BA secretion disorders in the liver, blood BA levels increased significantly, and an increased BA reflux rate causes the increase in TBA levels in ileum [14]. FXR-based regulation of BAs is effective in the treatment of liver injury.

Studies have shown that elevated transaminases and serum bilirubin may present with obstructive jaundice when the left and right hepatic ducts are obstructed at the same time or the common hepatic duct is obstructed, and patients may present with only elevated transaminases and normal serum total bilirubin when one hepatic duct is obstructed alone [18]. The detection results showed that serum AST, ALT, TBIL, Na^+^, and K^+^ contents in the control group were 118.4 ± 6.2 U/L, 55.7 ± 1.2 U/L, 1.9 ± 0.4 *μ*mol/L, 135.74 ± 4.76 mmol/L, and 4.14 ± 0.52 mmol/L, respectively; the serum AST content in the study group before treatment was 146.3 ± 9.7 U/L, significantly higher than that in the control group, and the difference had a statistical significance (*P* *<* 0.05); after treatment, the serum AST content was 123.5 ± 4.9 U/L, significantly lower than that before treatment, and the difference had statistical significance (*P* *<* 0.05); the TBIL content was 1.8 ± 0.3 *μ*mol/L, significantly lower than 2.2 ± 0.5 *μ*mol/L before treatment, and the difference had statistical significance (*P* *<* 0.05). The decrease in transaminase and serum bilirubin in the patient's body suggested that the obstructive jaundice was effectively improved. This is similar to the results of a simulation experiment by Yan-Xi et al. [19]. The detection results of the changes of liver function in patients at different obstruction sites showed that after treatment, the serum ALT content of 55.7 ± 31.6 U/L, AST content of 66.4 ± 42.4 U/L, and TBIL content of 215.4 ± 136.32 *μ*mol/L in patients with high obstruction were significantly decreased compared with those before treatment; the differences had statistical significance (*P* *<* 0.05); the serum ALT content of 47.4 ± 32.8 U/L, AST content of 56.1 ± 25.9 U/L, and TBIL content of 142.5 ± 123.6 *μ*mol/L in patients with low obstruction were significantly decreased compared with those before treatment; the differences had statistical significance (*P* *<* 0.05).

The article "Magnetic Resonance Cholangiopancreatography to Evaluate Improvement Effect of FXR Regulating Bile Acid on Hepatocellular Carcinoma with Obstructive Jaundice" was published in 2022. Journal: Contrast Media Mol Imaging.

Diffusion is an irregular thermal movement process of water molecules, also known as Brownian motion, which can reflect the water molecule movement of human tissues and organs by measuring the ADC value, and then reflect the physiological and pathological characteristics of body tissue structure [20]. The results of MRI showed that ADC was 1.34 ± 0.32 × 10^−3^ mm^2^/s in the control group, 1.24 ± 0.44 × 10^−3^ mm^2^/s in patients with mild jaundice, 1.18 ± 0.67 × 10^−3^ mm^2^/s in patients with moderate jaundice, and 1.02 ± 0.66 × 10^−3^ mm^2^/s in patients with severe jaundice before treatment, and the difference was statistically significant compared with the control group, *P* *<* 0.05; ADC was 1.17 ± 0.49 × 10^−3^ mm^2^/s in patients with moderate jaundice and 1.20 ± 0.27 × 10^−3^ mm^2^/s in patients with severe jaundice after treatment, and the difference was statistically significant compared with that before treatment, *P* *<* 0.05. The possible mechanisms were analyzed as follows: (1) due to the increase in serum bilirubin, bile salts, and plasma endotoxin concentration, the apoptosis of hepatocytes was accelerated: the Na^+^-K^+^ ATPase activity of hepatocytes was inhibited, resulting in cytotoxic edema and bile duct. Bile duct epithelial proliferation and a small amount of irregular capillary network was formed around the new bile duct, which increased the cell density and decreased the intercellular space, limiting the diffusion movement of water molecules; (2) the role of increased pressure in the upper bile duct of obstruction and cytokines released by macrophages, bile duct epithelial proliferation, and capillary network formation around the new bile duct, so that the cell density increased and the intercellular space became smaller, further leading to limited water molecule diffusion; (3) cholestasis and inflammatory cell infiltration, resulting in liver microarchitecture destruction and remodeling, caused microcirculatory pathway disorders, intrahepatic microthrombosis, and reduced hepatic effective blood flow, resulting in decreased measured ADC values. However, although the ADC values of patients with mild jaundice increased slightly, there was no significant difference compared with those before treatment, with no statistical significance, *P* *>* 0.05. It may be because in mild jaundice, after obstruction, the serum bilirubin level was slightly increased, the pressure in the bile duct was increased, the bile canaliculi were dilated, the microvilli were reduced, the normal structure of desmosomes was destroyed, and the bile solute molecules in bile canaliculi diffuse or reflux to the surrounding, causing osmotic pressure changed; a large number of water molecules entered the intercellular space, resulting in increased intercellular space and increased diffusion movement of water molecules, which counteracted with the factors limiting the movement of water molecules and made the increased measured ADC value. When bilirubin continued to rise, factors that limited the movement of water molecules dominated, resulting in reduced ADC values.

The article "Magnetic Resonance Cholangiopancreatography to Evaluate Improvement Effect of FXR Regulating Bile Acid on Hepatocellular Carcinoma with Obstructive Jaundice" was published in 2022. Journal: Contrast Media Mol Imaging.

## 5. Conclusion

FXR inhibitor was used to regulate BA in the treatment of obstructive jaundice injury in liver cancer, and the therapeutic effect was detected by MRI cholangiopancreatography. The results showed that the regulation of BA based on FXR could regulate the reabsorption of BA, accelerate the circulation of BA, restore the homeostasis of BA metabolism, play a hepatoprotective role, reduce bilirubin content in the body, and improve jaundice injury, which has application value. However, due to the limitation of experimental conditions, the included sample size is small, there is no significant difference in the changes of some data, and the liver function is strong and the physiological and pathological changes are complex, resulting in that the measurement of the ADC value is affected. Therefore, it still needs to further expand the sample size for further study and confirmation.

## Figures and Tables

**Figure 1:** Basic information of patients.

**Figure 2:** Changes in the serum TBA content. ^∗^Compared with the control group, *P* *<* 0.05; #compared with that before treatment, *P* *<* 0.05.

**Figure 3:** Changes of the intrahepatic TBA content. ^∗^Compared with the control group, *P* *<* 0.05; #compared with that before treatment, *P* *<* 0.05.

**Figure 4:** Changes in various indexes of the liver function test. ^∗^Compared with the control group, *P* *<* 0.05; #compared with that before treatment, *P* *<* 0.05. (a) AST (U/L). (b) ALT (U/L). (c) TBIL (umol/L). (d) Na+ (mmol/L). (e) K+ (mmol/L).

**Figure 5:** Changes of liver function in patients with high obstruction. ^∗^Compared with that before treatment, *P* *<* 0.05.

**Figure 6:** Changes of liver function in patients with low obstruction. ^∗^Compared with that before treatment, *P* *<* 0.05.

**Figure 7:** Changes in the ADC value before and after treatment. ^∗^Compared with that before treatment, *P* *<* 0.05; #compared with the control group, *P* *<* 0.05.

**Table 1:** General information of patients.

Group	Cases	Age/years old	Male/cases	Female/cases
Study group	48	52.61 ± 9.59	20	28
Control group	10	46.74 ± 7.92	5	5

## Data Availability

The data used to support the findings of this study are available from the corresponding author upon request.
